The article "Targeted Inhibition of Protein Tyrosine Phosphatase 1B by Viscosol Ameliorates Type 2 Diabetes Pathophysiology and Histology in Diabetic Mouse Model" was published in 2022. Journal: Biomed Res Int.

# Targeted Inhibition of Protein Tyrosine Phosphatase 1B by Viscosol Ameliorates Type 2 Diabetes Pathophysiology and Histology in Diabetic Mouse Model

**DOI:** 10.1155/2022/2323078

**Published:** 2022-08-22

**Authors:** Aamir Sohail, Hajra Fayyaz, Hamza Muneer, Idrees Raza, Muhammad Ikram, Zia Uddin, Sarah Gul, Hailah M. Almohaimeed, Ifat Alsharif, Fatima S. Alaryani, Imran Ullah

**Affiliations:** ^1^Department of Biochemistry, Faculty of Biological Sciences, Quaid-i-Azam University, Islamabad 45320, Pakistan; ^2^Department of Pharmacy, COMSATS University Islamabad, Abbottabad Campus, Abbottabad, 22060 KP, Pakistan; ^3^Department of Biological Sciences, FBAS, International Islamic University, Islamabad, Pakistan; ^4^Department of Basic Science, College of Medicine, Princess Nourah Bint Abdulrahman University, P.O.Box 84428, Riyadh 11671, Saudi Arabia; ^5^Department of Biology, Jamoum University College, Umm Al-Qura University, 21955 Makkah, Saudi Arabia; ^6^College of Science, Department of Biology, University of Jeddah, Jeddah, Saudi Arabia

## Abstract

Type 2 diabetes mellitus (T2DM) is one of the most common forms of diabetes. We are living in the middle of a global diabetes epidemic. Emerging pieces of evidence are suggesting the increased expression of protein tyrosine phosphatase 1B (PTP1B) in the pancreas and adipose tissues during T2DM. The negative regulation of the insulin signaling pathway by PTP1B helps the researchers to consider it as a potential therapeutic target for the treatment of insulin resistance and its associated complications. From the literature, we found that compound 5,7-dihydroxy-3,6-dimethoxy-2-(4-methoxy-3-(3-methyl-2-enyl)phenyl)-4H-chromen-4-one (Viscosol) extracted from Dodonaea viscosa can inhibit PTP1B in vitro. Therefore, in this study, we aimed to evaluate the antidiabetic effect of this compound in a high-fat diet (HFD) and low-dose streptozotocin- (STZ-) induced T2DM mouse model. For this purpose, T2DM was induced in C57BL/6 male mice by using an already established protocol with minor modification. The compound-treated T2DM mice showed improvements in biochemical parameters, i.e., decrease in the fasting blood glucose level, increased body weight, improved liver profile, and reduction in oxidative stress. Furthermore, to elucidate the inhibition of PTP1B, the expression level of PTP1B was also measured at mRNA and protein levels by real-time PCR and western blot, respectively. Additionally, downstream targets (INSR, IRS1, PI3K, and GLUT4) were examined for confirming the inhibitory effect of PTP1B. Our results suggest that the compound can specifically inhibit PTP1B in vivo and might have the ability to improve insulin resistance and insulin secretion. Based on our experiment, we can confidently state that this compound can be a new PTP1B drug candidate for the treatment of T2DM in the coming future.

The article "Targeted Inhibition of Protein Tyrosine Phosphatase 1B by Viscosol Ameliorates Type 2 Diabetes Pathophysiology and Histology in Diabetic Mouse Model" was published in 2022. Journal: Biomed Res Int.

## 1. Introduction

T2DM is a disorder characterized by chronic hyperglycemic condition and appears as one of the defining medical challenges of the 21st century. According to the International Diabetes Federation (IDF) Atlas of Diabetes (2021), currently, 537 million individuals are living with diabetes. Pakistan has 33 million reported cases of diabetes and has a comparative prevalence of 30.8%, and an increase up to 33.6% in 2045 is expected, while a 46% increase is expected to occur globally [1]. About 90-95% of diabetes cases are T2DM [2]. It is a complex metabolic disorder, described with the increase in blood glucose level caused by the dysfunction in pancreatic *β* cells which leads to defective insulin signaling and secretion [3]. This type of diabetes is also known as non-insulin-dependent diabetes mellitus and is described as the combination of hyperglycemia, insulin deficiency, and insulin resistance [4], and this combinatory condition causes impairment to a number of the systems in the human body, i.e., immune, musculoskeletal, neurological, and vascular. Numerous drugs are available for the treatment of T2DM but have several side effects and implications such as weight gain, cardiovascular problems, hypoglycemia, and gastrointestinal problems. Therefore, there is a need to find a solution for T2DM which would have fewer side effects [5]. The insulin signaling pathway starts as the insulin (INS) binds with the insulin receptors (IR). The autophosphorylation of IR leads to the recruitment of insulin receptor substrate (IRS); further downstream phosphorylation of IRS1/2 results in the activation of the combinatorial possibility of the pathway IR–IRS1/2–PI3K–Akt. Akt is also called Protein Kinase B (PKB). The activation of Akt leads to the translocation of GLUT-4 [6], while the translocation of GLUT4 from the cytoplasm to the plasma membrane handles transferring more glucose inside the cell to minimize the glucose level in blood [7]. Insulin signaling is regulated at several steps as cellular phosphatases are involved in attenuating the insulin signaling by dephosphorylating the insulin receptor which is activated by autophosphorylation [8]. PTP1B, a member of the PTP superfamily, is a major nontransmembrane PTP, encoded by the Ptpn1 gene and ubiquitously expressed in all tissues [9]. PTP1B has a C-terminal hydrophobic region which anchors the protein to the cytoplasmic face of the endoplasmic reticulum and facilitates its ability to substrates. PTP1B inhibits insulin signaling by dephosphorylating the tyrosine residues of IRS-1 and IR-*β* [10]. The PTP1B is highly expressed in tissues that regulate glucose metabolism, i.e., the heart, skeletal muscles, pancreatic *β* cells, and liver [11]. In recent years, PTP1B has been the center of focus because of its ability to attenuate the insulin signaling pathway and is currently considered a therapeutic target against diabetes. The negative regulation of insulin metabolism via PTP1B is already demonstrated by using tissue-specific (liver) and whole-body PTP1B knockout mice. It is well-known that inhibition of PTP1B can reduce insulin insensitivity hence increasing glucose uptake [12, 13]. Dephosphorylation of insulin receptors by PTP1B is reported both in vitro as well as in vivo. Furthermore, an increase in the expression of PTP1B causes insulin resistance in the liver, adipose, and muscle tissues [14–16]. Dodonaea viscosa (L). Jacq, a member of the family Sapindaceae grows on rocky and poor soils, is an evergreen shrub. Dodonaea viscosa is centrally originated in Australia and is also distributed in Mexico, Africa, New Zealand, India, Northern Mariana Islands, Virginia Islands, Florida, Arizona, South America, and Pakistan [17]. Extracts from the Dodonaea viscosa showed antidiabetic effects in alloxan and streptozotocin-induced diabetes in animal models [18, 19]. In 2010, Veerapur et al. reported the antidiabetic, antioxidant, and hypolipidemic activity of the aerial parts of Dodonaea viscosa in the streptozotocin-induced diabetes rat model [20]. Several studies have confirmed the antimicrobial, anti-inflammatory, antiulcer, smooth muscle relaxant, and wound healing activity of this plant [21]. Rojas et al. screened 294 plants and identified the hypoglycemic activity of Dodonaea viscosa [22]. Dodonaea viscosa is a major source of PTP inhibitors, as revealed by Ziauddin et al. in 2018. They were able to identify a purified polyphenolic compound from aerial parts of the plant which was showing an antidiabetic effect. This potent bioactive compound was isolated as a pale-yellow solid (molecular formula C_23_H_24_O_7_), with a molecular weight of 412.1522. Overall, they have isolated 9 compounds and all compounds have an IC_50_ value of 13.5-57.9 *μ*M. However, the compound 4, (5,7-dihydroxy-3,6-dimethoxy-2-(4-methoxy-3-(3-methyl but-2-enyl)phenyl)-4H-chromen-4-one), a potent inhibitor of PTP1B has an IC_50_ value of 13.5 *μ*M and exhibits more fold inhibitory activity than other isolated compounds [23]. It was also inferred from the analysis that this compound works by the mechanism of mixed type 1 inhibition in vitro. In the current study, diabetes was induced by feeding mice with a high-fat diet and carbohydrates resulting in increased plasma insulin levels causing glucose intolerance and insulin resistance. The mice were further followed by a streptozotocin injection causing *β* cell death and a decrease in *β* cell mass [24]. Furthermore, we have designed our study to explore the insulin signaling pathway in the presence of compound 4, and the obtained results suggested that the compound was able to block PTPB1. This inhibition also enhances the secretion of insulin and glucose metabolism by increasing the GLUT4 translocation.

The article "Targeted Inhibition of Protein Tyrosine Phosphatase 1B by Viscosol Ameliorates Type 2 Diabetes Pathophysiology and Histology in Diabetic Mouse Model" was published in 2022. Journal: Biomed Res Int.

## 2. Materials and Methods

### 2.1. Animals and Grouping

C57BL/6 mice (25-40 g, 8-12 weeks old), purchased from the National Institute of Health (Islamabad, Pakistan), were used in the current study. Animals were maintained in the animal facility of Quaid-i-Azam University according to the guidelines of the National Institute of Health (USA) and the bioethics committee of our university. All protocols for animal handling and experimentation were approved by the Institutional Review Board. The mice were divided into three separate groups (*n* = 3 in each group): group 1, control as a positive control; group 2, STZ-HFD-induced diabetic; and group 3, STZ-HFD compound-treated group.

### 2.2. Induction of Diabetes and Compound Treatment

The control group was fed the standard diet (4.1% fat, 22.2% protein, and 12.1% carbohydrates, as a percentage of total kcal) and injected with a single 500 *μ*L injection of saline. For diabetes induction, all the mice fasted for 4-6 hours before the injection of STZ, and blood glucose level (BGL) was estimated by a glucometer (ACCU-CHEK Instant S, Roche Diagnostic, Mannheim, Germany). Diabetes was induced by intraperitoneal injection of streptozotocin (Bio plus Fine Research Chemical, CAT # 41910012-3, Bioworld) for 5 consecutive days at a dose of 40 mg/kg in 500 *μ*L saline. The STZ injected mice were fed on a high-fat diet (HFD, 58% fat, 25% protein, and 17% carbohydrate, as a percentage of total kcal) with 10% glucose solution. On the sixth day, mice were given, and it took around 9-10 days for mice to develop diabetes. Mice with fasting blood glucose levels of >250 mg/dL (>11.1 mM) were considered diabetic. The BGL was continuously checked by a glucometer until euthanized. In group 3, after the induction of diabetes, HFD was removed. On the 11th day, the compound (5,7-dihydroxy-3,6-dimethoxy-2-(4-methoxy-3-(3-methyl but-2-enyl)phenyl)-4H-chromen-4-one) was dissolved in 1% dimethyl sulfoxide (DMSO), and a single intraperitoneal injection (500 *μ*L) was given to mice (33 mg/kg). After the treatment with the compound, the BGL of the mice was continuously checked for 7 days. On the 17th day after BGL estimation, mice were euthanized for further analysis.

The article "Targeted Inhibition of Protein Tyrosine Phosphatase 1B by Viscosol Ameliorates Type 2 Diabetes Pathophysiology and Histology in Diabetic Mouse Model" was published in 2022. Journal: Biomed Res Int.

### 2.3. Serum Blood Glucose Analysis

The fasted mice for 4-6 hours were used to check the blood glucose level during the whole study. For output, blood was obtained through the tail vein, and glucose level was checked using a glucometer (ACCU-CHEK Instant S).

### 2.4. Blood Collection and Serum Separation

At the end of the study, mice were anesthetized, and blood was collected by cardiac puncture with the help of a 23G needle. Serum was separated in 4 mL gel and clot activator vacutainer (Xinle) by centrifuging the tubes at 6000 rpm for 10 min. The supernatant was collected, and sera were stored at -20°C until further use.

### 2.5. Biochemical Parameters

The antidiabetic effects of the compound in HFD-STZ-induced diabetes in mice were seen. Different biochemical parameters were analyzed. These assays were performed by using enzymatic kits bought from AMP diagnostics. All the procedures and methods performed were according to the given protocol of kits.

#### 2.5.1. Liver Profiling

Liver function biomarkers, including alanine aminotransferase (ALT), aspartate aminotransferase (AST), and alkaline phosphatase (ALP), were assayed by using a commercially available liver profiling kit (AMP Diagnostics, Austria).

#### 2.5.2. ROS Assay

For ROS assay, according to Hayashi et al., protocol was followed for estimating the ROS levels in the serum of mice. Hydrogen peroxide was used as the standard solution and incubated at 37°C after 5 min. The working buffer was prepared according to the protocol by adding 100 *μ*L of R1 and R2 buffers. The working buffer was added at a ratio of 1 : 25 and incubated at 37°C for 1 min. Afterward, absorbance was measured by a multiskan GO, spectrophotometric plate reader (Thermo Fisher Scientific, USA) spectrophotometer at 505 nm. Three readings were recorded at 505 nm at an interval of 15 seconds. A calibration curve was constructed by using the concentration of hydrogen peroxide, and, respectively, samples were analyzed according to that [25].

### 2.6. Histological Analysis by H&E Staining

The liver and pancreas were removed and flushed with PBS and distilled water. The organs were fixed in 10% formalin and kept at room temperature. For histological studies, these organs were then removed, dehydrated, and embedded in the paraffin wax. The fixed tissues were sectioned (4 *μ*m) using a microtome (KD202, China). The tissue sections were stained with hematoxylin and eosin stains. The stained slides were then examined under the bright field microscope (CX41, Olympus Microscope, Japan). ImageJ was used for image analysis and graphical representation of H&E staining.

The article "Targeted Inhibition of Protein Tyrosine Phosphatase 1B by Viscosol Ameliorates Type 2 Diabetes Pathophysiology and Histology in Diabetic Mouse Model" was published in 2022. Journal: Biomed Res Int.

### 2.7. RNA Isolation, cDNA Synthesis, and Real-Time qPCR

RNA was extracted from the respective tissues by using the RNA Extraction Kit (PureLink TM, RNA Minikit, Invitrogen by Thermo Fisher Scientific, Cat No # 1218301 8A). Approximately, 30-40 mg of tissue was used for the isolation of total RNA. Isolated RNA (1 *μ*g) was reverse transcribed to cDNA using a high-capacity cDNA synthesis kit (Thermo Fischer Scientific, RevertAid First Strand cDNA Synthesis Kit, USA). The relative abundance of mRNA levels was measured by SYBER Green-based RT-PCR chemistry (Maxima SYBR Green/ROX qPCR Master Mix (2X), Thermo Scientific, USA) using the MyGo Pro PCR system (MyGo PCR systems, IT-IS Life Sciences). Specific primers were used for RT-PCR (Table 1). Each sample was run in triplicates, and *β*-actin was used as a housekeeping gene. The data were analyzed by the *ΔΔ*Ct method, and mRNA fold change was calculated.

### 2.8. Western Blotting

For western blotting, whole-cell lysate was prepared by using radioimmunoprecipitation assay (RIPA) buffer (10 mM Tris pH 8, 140 mM NaCl, 1% Triton X-100, 0.1% SDS, 0.01% sodium deoxycholate, 1 mM EDTA, 1 mM DTT, 1% protease inhibitor, 1% phosphate inhibitor). Depending upon the size of the tissue (20-30 mg), the 200-300 *μ*L buffer was added to a tube having tissue and was minced. The samples were incubated on ice for 15 minutes and vortexed at intermittent intervals of 15 seconds. The samples were additionally incubated on ice for 15 minutes. The whole-cell lysate was centrifuged at 4°C at maximum speed (13000 rpm) for 10 minutes. The supernatant was pipetted out and stored at -20°C for future use. The isolated protein was quantified by Bradford assay using BSA. The concentration of unknown protein samples was figured out from the standard curve by applying the trendline formula of MS Excel. GAPDH was used as a loading control. The data of immunoblotting was analyzed by software (AlphaView SA version 3.4.4.0), and integrated optical density was calculated.

### 2.9. Statistical Analysis

For statistical analysis, data from at least three replicates were used and analyzed with a one-way, two-way ANOVA, and post hoc Tukey or LSD test using GraphPad Prism (version 9). Microsoft Excel was used for *ΔΔ*Ct calculation. A *p* value of < 0.05 was considered statistically significant. All experiments were performed in triplicates.

## 3. Results

### 3.1. Mean Body Weight and Fasting Blood Glucose Level

Bodyweight and blood glucose levels (BGL) were monitored during the experimental period in all three groups. STZ-HFZ compound-treated group showed improvements in body weight as compared to the STZ-HFD-induced diabetic group (diabetic) (Figure 1). In STZ-HFD compound-treated group, a gradual decrease in the BGL was seen after the treatment with a single injection of the compound (Figure 2), while BGL levels in STZ-HFD-induced group remained constantly high.

The article "Targeted Inhibition of Protein Tyrosine Phosphatase 1B by Viscosol Ameliorates Type 2 Diabetes Pathophysiology and Histology in Diabetic Mouse Model" was published in 2022. Journal: Biomed Res Int.

### 3.2. Biochemical Parameters

Biochemical testing was performed using the serum. In diabetes, liver damage and alteration in liver enzymes were seen. Hence, liver profiling was performed by analyzing the level of AST, ALT, and ALP enzymes. The level of AST, ALT, and ALP was significantly higher in the STZ-HFD-induced group as compared to normal and STZ-HFD compound treated (Figure 3). Moreover, the compound showed a liver protective effect as the level of AST, ALT, and ALP was comparable to the control group. The absorbance was measured at 340 nm, and analyzed data were represented in the form of a bar graph. Furthermore, ROS level was analyzed in the serum which was found significantly low in the STZ-HFD compound-treated group compared to STZ-HFD-induced group (Figure 4).

### 3.3. Histological Analysis by H&E Staining

The liver of the STZ-HFD-induced group showed abnormal patterns with lymphocyte infiltration, lobular inflammation, hyperammonemia, and various spots of cytoplasmic degeneration. However, the morphology of the STZ-HFD compound-treated group was like the control group with slight lymphocyte infiltration and liver regeneration (Figure 5(a)). In the case of the liver, the area was selected by using ImageJ, and cells were analyzed. The obtained value was exported to excel for analysis. The selected area obtained from the STZ-HFD-induced and STZ-HFD compound-treated groups was normalized by the control group. The relative number of the normal cell in the liver (Figure 5(b)) and inflammatory lobules in the liver (Figure 5(c)) was represented in the form of a bar graph. Significant results were found with one-way ANOVA, with a *p* value < 0.0001.

In the pancreas, the control and STZ-HFD compound-treated groups showed similar morphology as compared to STZ-HFD-induced group; as the pancreatic morphology was distorted, inflammatory cell invasion and reduction in the *β* cell mass were seen (Figure 6(a)). In the case of the pancreas, the area was selected by using ImageJ, and cells were analyzed. The obtained value was exported to Excel for analysis. The selected area obtained from the STZ-HFD-induced and STZ-HFD compound-treated groups was normalized by the control group. The relative number of the normal cell in the pancreas (Figure 6(b)) and inflammatory lobules in the pancreas (Figure 6(c)) was represented in the form of a bar graph. Significant results were found with one-way ANOVA, with a *p* value < 0.0001.

The article "Targeted Inhibition of Protein Tyrosine Phosphatase 1B by Viscosol Ameliorates Type 2 Diabetes Pathophysiology and Histology in Diabetic Mouse Model" was published in 2022. Journal: Biomed Res Int.

### 3.4. Correlation of Inhibition of PTP1B in Adipose and Pancreas with the Expression of Downstream Regulators

PTP1B is widely expressed in insulin-sensitive tissues and plays a role as an important negative regulator of insulin signaling. Many studies have reported that inhibition of PTP1B can be considered a therapeutic target in T2DM. Therefore, we further investigated the expression of different downstream components in both tissue (adipose and pancreas) as possibly the inhibition of PTP1B is a contributing factor to insulin signaling. Each cDNA sample was run in triplicates, and GAPDH was used as a housekeeping gene. The data from three independent experiments were analyzed by a *ΔΔ*Ct method to calculate the mRNA fold change using normal as a control. The data were represented as means ± SD. The differences between groups were analyzed by two-way ANOVA using Bonferroni post hoc test. A *p* value of 0.05 was considered statistically significant. Our data showed that the relative abundance of PTPN1 mRNA, the main unit of our study, was decreased in the treated group in both tissues (Figures 7(a) and 8(a)). Moreover, it is known that PTPN1 inhibits the phosphorylation of IR and IRS1. Therefore, inhibition of PTPN1 results in increased expression of INSR, IRS1, PI3K, and GLUT4 in adipose (Figures 7(b)–7(e)) and INS, IRS1, and PI3K in the pancreas (Figures 8(b)–8(d)) in the compound-treated group as compared to the STZ-HFD diabetic group. Hence, we can conclude that inhibition of PTP1B results in the reduction of mRNA level of PTPN1 which increased downstream regulatory components of insulin signaling. These results show that the compound used during the study can block the activity of PTPN1 at the mRNA level which affects the components of insulin signaling.

### 3.5. Immunoblotting Showing the Expression of PTP1B and Insulin in Adipose Tissue

To further substantiate the RT-qPCR results, the expression of PTP1B and insulin at the protein level was analyzed by immunoblotting in adipose tissue. The results showed that PTP1B was increased in the adipose tissue of the STZ-HFD-induced group while the reduction in the expression was seen in the compound-treated group (Figure 9(a)). Furthermore, lower expression of insulin was found in the STZ-HFD-induced group, while in the control and compound-treated groups, significant insulin secretion was detected (Figure 9(b)). The immunoblot was analyzed by software (AlphaView SA version 3.4.4.0), and the bar graph is plotted by calculating the integrated optical density (IOD) value by ImageJ. IOD of targets was normalized with GAPDH as an internal control (Figures 9(c)–9(e)). Significant results were found with one-way ANOVA, as ∗∗∗*p* = 0.0008.

The article "Targeted Inhibition of Protein Tyrosine Phosphatase 1B by Viscosol Ameliorates Type 2 Diabetes Pathophysiology and Histology in Diabetic Mouse Model" was published in 2022. Journal: Biomed Res Int.

## 4. Discussion

Type 2 diabetes mellitus is regarded as resistance to insulin hormone which occurs because of attenuated signaling from the insulin receptors. The global occurrence of T2DM is increasing at an alarming rate. Protein tyrosine phosphatase 1B (PTP1B), a member of PTPase, has been getting intensive attention in research as it takes part in the insulin signaling cascade. The compelling experiments have revealed that PTP1B plays a significant regulatory role in modulating insulin sensitivity, hence, signifying PTP1B as a potential therapeutic target. PTP1B is not only involved in T2DM but also involved in several other diseases, including autoimmune disorders, cardiovascular diseases, cancer, and liver diseases.

Several pieces of evidence from cellular, biochemical, and chemical inhibitor studies have found that PTP1B is a major negative regulator of insulin signaling. Additionally, many studies suggest that the action of insulin can be enhanced by the inhibition of PTP1B. Subsequently, PTP1B has been considered an attractive target for the treatment of T2DM. In the present study, we tried to analyze the PTP1B inhibitory role of our specific compound extract from Dodonaea viscosa in *vivo*. Our findings highlight the intriguing fact that inhibition of PTP1B might help to improve insulin resistance and insulin secretion in adipose and pancreatic tissue. Improvements in biochemical parameters such as the decrease in the fasting blood glucose level, increased body weight, and improved liver profile were also seen in our experiment which is consistent with the previously published reports [26]. Histopathological analysis by H&E staining of the liver and pancreas showed comparable results of the STZ-HFD compound-treated and normal groups, while the morphology of liver and pancreas was distorted in the STZ-HFD diabetic group as lymphocyte infiltration, reduced *β* cell mass, and apoptotic cells were seen. In recent years, *in vitro* analysis has shown that PTP1B expression can be induced by high glucose, palmitate, fatty acids, and cytokines such as TNF-*α* and IL-6 [11, 27–29]. The increased level of PTP1B is reported in insulin-sensitive tissues in STZ-induced diabetic mice and rats [30]. In 2012, Vakili et al. reported that inhibiting PTP1B by using shRNA in STZ-induced diabetic mice resulted in a decrease in plasma glucose level [31]. Furthermore, our study also shows a significant reduction in oxidative stress. The elevated level of reactive oxygen species (ROS) in obesity and diabetic individuals has been previously reported [32]. Likewise, in the current study, the level of ROS in the STZ-HFD-induced group was significantly high than in the STZ-HFD compound-treated group which confirms the protective effect of our compound.

The article "Targeted Inhibition of Protein Tyrosine Phosphatase 1B by Viscosol Ameliorates Type 2 Diabetes Pathophysiology and Histology in Diabetic Mouse Model" was published in 2022. Journal: Biomed Res Int.

It has been previously reported that PTP1B inhibitors increased the IR and IRS1 phosphorylation which results in the increased GLUT4 translocation and glucose uptake in insulin target tissues [33]. Several studies also showed that PTP1B deficient animals enhanced insulin sensitivity, prevented them from weight gain, and increased phosphorylation of IR even if they are fed with an HFD [34]. Likewise, our study also shows that there would be an increased translocation of glucose via GLUT4 which ultimately upregulate the insulin signaling pathway. This phenomenon was confirmed by analyzing the relative mRNA expression of *INS*, *INSR*, *IRS1*, *PI3K*, *GLUT4*, and *PTPN1*. In adipose tissue, we found that the relative mRNA expression of *INSR*, *IRS1*, *PI3K*, and *GLUT4* was downregulated in the STZ-HFD diabetic group while upregulated in the STZ-HFD compound-treated group. Furthermore, expression of *PTPN1* was significantly decreased in the compound-treated group. Similarly, we have seen an increased expression of *INS* and *IRS1* in the compound-treated group, while downregulation of *PTPN1* in pancreatic tissues which were found consistent with the previously reported studies [10].

To substantiate our results, we have confirmed the expression of PTP1B and insulin at the protein level in adipose tissue. We found increased expression of PTPN1 in the STZ-HFD-induced group, while it was inhibited in the compound-treated group. The antidiabetic activity of Dodonaea viscosa (plant extract) is well-known and observed for many years, but a lead compound that can inhibit the PTP1B enzyme was yet not explored. Hence, this assures us that the compound used in the current study can be considered a specific inhibitor of PTP1B.

## 5. Conclusion

Concluding, we have targeted PTP1B and its downstream targets in the STZ-HFD-induced type II diabetic model via the help of a compound, 5,7-dihydroxy-3,6-dimethoxy-2-(4-methoxy-3-(3-methyl-2-enyl)phenyl)-4H-chromen-4-one, extracted from the Dodonaea viscosa. The antidiabetic and inhibitory potential of this compound on PTP1B has been evaluated in the current study. Collectively, we have investigated the effect of our compound on body weight, histological, and biochemical parameters. Additionally, the study was supported by transcriptomic and proteomic analyses. The data shows a decrease in the level of PTP1B at the mRNA level, and complete inhibition was seen in the compound-treated group. Conclusively, this study will help to develop a new pharmacological drug for the treatment of T2DM specifically by targeting PTP1B.

The article "Targeted Inhibition of Protein Tyrosine Phosphatase 1B by Viscosol Ameliorates Type 2 Diabetes Pathophysiology and Histology in Diabetic Mouse Model" was published in 2022. Journal: Biomed Res Int.

## Figures and Tables

**Figure 1:** Mean body weight (g) of all groups of mice versus experimental days. The normal group was only given a standard diet, while STZ-HDF induced and STZ-HFD compound treated were given 5 I.P. STZ injections. Ordinary two-way ANOVA was performed, and results were found significant, ^∗∗∗∗^*p* < 0.0001.

**Figure 2:** Mean blood glucose level (BGL). The bar graph showing increased BGL in the STZ-HFD-induced group as compared to the control group. While a significant reduction was observed in the compound-treated group as compared to diabetic, two-way ANOVA was used for calculating the statistical significance; ^∗∗^*p* < 0.001.

**Figure 3:** Serum enzymatic activities (U/L) of liver function (AST, ALT, and ALP) in mice. The bar graph showing the levels of AST, ALT, and ALP which was elevated in the STZ-HFD-induced group as compared to the control group. And significant reduction was observed in the compound-treated group as compared to diabetic. Two-way ANOVA was used for calculating the statistical significance; ^∗∗∗∗^*p* < 0.0001.

**Figure 4:** Serum ROS level. ROS level was elevated in the STZ-HFD-induced group as compared to the control and treated groups. Two-way ANOVA was used for calculating the statistical significance; ^∗∗∗^*p* < 0.0531.

**Figure 5:** (a) H&E staining of liver tissue at 10x. Normal control, no significant change was seen in the morphology of the liver. STZ-HFD-induced diabetic mice, representing tissue damage, necrosis at many spots, and lymphocyte infiltration. STZ-HFD compound treated, the image was comparable to the normal with slight inflammatory invasion and tissue regeneration. Here, arrow represents lobular inflammation and cell invasion, star represents hyperaemia, and triangle represents cellular degeneration. (b) The area was selected by using ImageJ, and cells were analyzed. The number of the normal cell was represented in the form of a bar graph. Significant results were found with one-way ANOVA, as ^∗∗∗^*p* = 0.5483. (c) The inflammatory lobules were represented in the form of a bar graph. Significant results were found with one-way ANOVA, as ^∗∗∗^*p* = 0.3272.

**Figure 6:** (a) H&E staining of pancreatic tissues. The images are obtained from a bright field microscope at 40x. Normal control with normal pancreatic structure. STZ-HFD-induced diabetic with damaged pancreatic tissue reduced *β* cell mass and inflammatory cell invasion. STZ-HFD compound treated having a structure comparable to the normal group. Here, upper arrow represents inflammatory lobules and cells, and arrow represents a reduction in *β* cell mass. (b) The area was selected by using ImageJ, and cells were analyzed. The number of normal cell was represented in the form of a bar graph. Significant results were found with one-way ANOVA, as ^∗∗∗^*p* = 0.2058. (c) The inflammatory lobules were represented in the form of a bar graph. Significant results were found with one-way ANOVA, as ^∗∗∗^*p* = 0.1526.

The article "Targeted Inhibition of Protein Tyrosine Phosphatase 1B by Viscosol Ameliorates Type 2 Diabetes Pathophysiology and Histology in Diabetic Mouse Model" was published in 2022. Journal: Biomed Res Int.

**Figure 7:** Expression profile of PTPN1 and downstream component of insulin signaling in mouse adipose tissue reveal significant difference. (a–e) The bar graphs show relative abundance of PTPN1, INSR, IRS1, PI3K, and GLUT4 mRNAs presented as fold change using control group as a reference sample. *n* = 3 mice. Two-way ANOVA test was used for calculating the statistical significance; ^∗∗∗^*p* < 0.05.

**Figure 8:** Expression profile of PTPN1 and downstream component of insulin signaling in mouse pancreatic tissue reveal significant difference. (a–d) The bar graphs show relative abundance of PTPN1, INS, IRS1, and PI3K mRNAs presented as fold change using control group as a reference sample. *n* = 3 mice. Two-way ANOVA test was used for calculating the statistical significance; ^∗∗∗^*p* < 0.05.

**Figure 9:** Immunoblotting reveals the expression of PTP1B and insulin in adipose tissue. The immunoblot (a, b) shows the expression of PTP1B and insulin. GAPDH was used as a loading control (c). The bar graph is plotted by calculating integrated optical density (IOD) value (d, e). It shows an increase in the expression of insulin and a decrease in PTP1B. We found significant results with one-way ANOVA, ^∗∗∗^*p* = 0.0008.

**Table 1:** List of primers used in RT-qP.

No.	Primer name	Sequence (5′ →3′)	Tm	Amplicon size
1	mPdx1-F	ACTTGAGCGTTCCAATACGG CTTAGCTTGCTCAGCCGTTC	60.1	85 bp
	mPdx1-R		60.3	
2	mIrs1-F	AAGCACTGTGACACCGGAA CTTCGTGACCAGCTGTCCTT	60.3	72 bp
	mIrs1-R		60.4	
3	mGlut4-F	ACATACCTGACAGGGCAAGG TGGAGGGGAACAAGAAAGTG	60	110 bp
	mGlut4-R		60.1	
4	mPi3k-F	GAGACAGGATGGGTCAAGGA CAAAGCAACACAGGAGAGCA	60	132 bp
	mPi3k-R		60.2	
5	mPtpn1-F	GCATAGGACAGTGGTAATGCG AACTCACAGGGAAAGCAGAGG	60.5	123 bp
	mPtpn1-R		60.8	
6	mInsr-F	CCTGTGGAGGGCTAACTGTG GGTTTGATACGGTGGAGGC	60.7	76 bp
	mInsr-R		60.3	
7	mInsulin-F	GCCAAACAGCAAAGTCCAG CACTAAGGGCTGGGGGTTA	59.4	85 bp
	mInsulin-R		59.9	
8	m*β*-actin-F	GATCATTGCTCCTCCTGAGC ACATCTGCTGGAAGGTGGAC	60	83 bp
	m*β*-actin-R		60	

## Data Availability

Our data will be available upon the publication of this manuscript.

## Abbreviations

IRS: Insulin receptor substrate
STZ: Streptozotocin
PTP1B: Protein-tyrosine phosphatase 1B
TCPTP45: T cell protein tyrosine phosphatase 45
Akt: Ak strain transforming
T2DM: Type 2 diabetes mellitus
AST: Serum aspartate aminotransferase
ALT: Serum alanine aminotransferase
ALP: Serum alkaline phosphatase
ROS: Reactive oxygen specie
b.w: Bodyweight
HFD: High-fat diet
PKB: Protein kinase B
IR: Insulin receptor
DMSO: Dimethyl sulfoxide.
